The article "Vesicle-Associated Membrane Protein-Associated Protein A Is Involved in Androgen Receptor Trafficking in Mouse Sertoli Cells" was retracted in 2019. Reasons: concerns about the data; concerns about the images; concerns about the results or conclusions.

# Vesicle-Associated Membrane Protein-Associated Protein A Is Involved in Androgen Receptor Trafficking in Mouse Sertoli Cells

**DOI:** 10.1155/2018/4537214

**Published:** 2018-03-04

**Authors:** Qiong Deng, Jianwen Zhang, Zhu Wang, Shengping Zhang, Fan Zhi, Hui Liang

**Affiliations:** Department of Urology, The People's Hospital of Longhua, Shenzhen, China

## Abstract

Androgen and its receptor (AR) play an important role in maintaining spermatogenesis and male fertility. The nonclassical androgen signaling pathway is proposed to be mediated by an AR in plasma membrane in Sertoli cells. Our previous studies showed that testosterone induces cytoplasmic AR translocation to plasma membrane by binding with caveolin-1. This study was conducted to the underlying molecular mechanism mediating AR trafficking. Data from mass spectrometry using membrane coimmunoprecipitation sample by anti-AR antibody indicated VAPA is a candidate protein. Knockdown of VAPA by shRNA decreased the amount of AR localized to membrane and nuclear fraction and prevented AR trafficking after being exposed to testosterone. Further studies indicated AR trafficking in Sertoli cells might be mediated by VAPA via association with vesicle transport protein OSBP. This study can enrich the mechanism of the androgen actions and will be helpful for further clarifying the nonclassical signaling pathway of androgens in Sertoli cells.

## 1. Introduction

Androgen and its receptor (AR) play an important role in maintaining spermatogenesis and male fertility. Evidences showed that the actions of androgen in Sertoli cells were essential for the proceeding of spermatogenesis. Sertoli cell-selected *AR* knockout mice exhibit spermatogenesis arrest at the diplotene stage [1–3], similar to the phenotype of *AR* knockout mice. The selected *AR* knockout in germ cells does not affect the process of the spermatogenesis [4]. These data suggested that the AR in Sertoli cells is critical of spermatogenesis.

AR associates with testosterone, and the complex translocates to nucleus, binds with the androgen response element (ARE) in the chromatin, and then induces gene transcriptional repression or activation. This is the classical pathway of androgen, taking several hours since it requires new protein synthesis and secretion. Compared with the classical pathway, a faster action of androgen called nonclassical signaling pathway was found. It only takes several seconds to minutes to response since it does not relate to DNA amplification or protein synthesis. And evidences suggested this fast action is mediated by a membrane receptor of androgens. Our previous data showed AR localized in the membrane of murine testicular TM4 cells, and testosterone enhanced the membrane association, AR localizes to plasma membrane by binding to Caveolin-1 [5, 6]. However, the precised mechanism mediating AR trafficking to the membrane remains unclear.

The article "Vesicle-Associated Membrane Protein-Associated Protein A Is Involved in Androgen Receptor Trafficking in Mouse Sertoli Cells" was retracted in 2019. Reasons: concerns about the data; concerns about the images; concerns about the results or conclusions.

In this study, we used coimmunoprecipitation (co-IP) and employed mass spectrograph (MS) to find the candidate protein involved in AR trafficking. The screened candidate proteins will be knock down using shRNA constructs to test the role in AR trafficking. We will also conduct experiments to study the molecular mechanism mediating AR trafficking by the candidate protein. This study will enrich the mechanism of the action of androgens and provide new sights into testosterone signaling pathway in Sertoli cells mediating spermatogenesis.

## 2. Materials and Methods

### 2.1. Reagents and Constructs

Unless otherwise indicated, all the chemical reagents were obtained from Sigma-Aldrich (USA), all of the cell culture reagents were bought from Life technologies (USA). The shRNA construct was provided by Shanghai Genechem Co. Ltd (China).

### 2.2. Cell Culture and Transfection

Murine Sertoli cell line TM4 was purchased from the American Type Culture Collection (ATCC, Manassas, VA). Cells were cultured in DMEM containing 10% FBS and 100 *μ*g/ml penicillin and 100 μg/ml streptomycin at 37°C. Cells plated in 10 cm culture dishes were transfected with shRNA or negative control using Lipofectamine 3000 (Invitrogen). Cells were changed to medium supplemented with stripped serum when reaching 80%–85% confluence. Eighteen hours later, the medium was changed to serum-free medium containing 0.1% BSA and incubated for 2 hours before exposure to 10 nM testosterone (Melone Pharma, China) for 30 minutes unless otherwise indicated.

### 2.3. Coimmunoprecipitation and Mass Spectrometry

Protein subcellular fractionation isolation was following the instruction provided in the kit as previously described [7]. 500–1000 *μ*g of protein was subjected to immunoprecipitation using 2.5 *μ*g of rabbit polyclonal antibody, anti-AR N-20 (Santa Cruz Biotechnology) and 2.5 *μ*g of rabbit polyclonal antibody, anti-AR (ab74272, Abcam). After separation of immunoprecipitated proteins using magnetic protein A/G Dynabeads (Invitrogen), pellets were washed by lysis buffer (containing 150 mM NaCl, 5 mM MgCl_2_, 2 mM EGTA, 50 mM Tris-HCl, and 1% Triton X-100) three times, 5 min each. Proteins were disassociated from the magnetic beads by incubating with 0.1 M glycine (pH 2.2–2.7) for 10 min. A part of co-IP samples was sent to FitGene Biotechnology Co. Ltd. (Guangzhou, China) for mass spectrometry (MS) detection and bioinformatic analysis, and the other was for Western blot analysis.

The article "Vesicle-Associated Membrane Protein-Associated Protein A Is Involved in Androgen Receptor Trafficking in Mouse Sertoli Cells" was retracted in 2019. Reasons: concerns about the data; concerns about the images; concerns about the results or conclusions.

### 2.4. Western Blot

Levels of proteins were measured using 20 *μ*g of protein or equal volume of co-IP samples. The samples were subjected to SDS-PAGE on 10% tricine-glycine gels and transferred onto polyvinyl difluoride membranes (Millipore). After blocking nonspecific protein-binding sites by incubation for 1 h at room temperature in TBST (Tris-buffered saline with 0.2% Tween 20) containing 5% nonfat dry milk, membranes were incubated overnight with primary antibody (antibodies information see Table 1). The membranes were washed with TBST for 5 min, repeated 3 times. Subsequently, the membranes were incubated with the secondary antibody in 5% nonfat dry milk at room temperature for 1 h. The specific complexes were detected using the enhanced chemiluminescence system from GE Healthcare. The densitometry of the bands was measured using software Image J.

### 2.5. Statistical Analysis

Data are represented as mean ± SEM. The statistical significance of the differences between groups was determined by one- or two-way ANOVA followed by Fisher protected least-significant difference posthoc test using software SigmaPlot. Statistical significance was set at *P* < 0.05.

## 3. Results

### 3.1. VAPA Is Identified as a Candidate Protein by MS

Agreeing with our previous studies [5, 6], Western blot data and statistical analysis showed testosterone induces cytoplasmic AR translocation to membrane fraction (Figure 1(a)). In order to clarify the molecular mechanism of AR translocation to membrane fraction, we used anti-AR antibody to immunoprecipitate the molecules in the membrane fraction that associated with AR. The co-IP experiment was verified by Western blot. The co-IP sample was running on a SDS gel, and silver staining showed multiple different bands. More co-IP samples were preloaded on the gels, and the sites with different bands were cut down, and sent to FitGene Biotechnology Co. Ltd. (Guangzhou, China) for MS detection.

As shown in Figure 1(b), in this site, five proteins (VAPA, ACTB, P5CR2, AXN1, and KRT) were identified. ACTB (Actin beta) and KRT (Keratin) were suggested as contaminated protein, since they were detected in most of the samples. P5CR2 (Pyrroline-5-carboxylate reductase 2) and AXN1 (Axin-1) were verified by co-IP and Western blot, and no positive data was observed (data not shown).

Vesicle-associated membrane protein-associated protein A (VAPA) presents in the plasma membrane and intracellular vesicles. This protein is reported in function in vesicle trafficking, membrane fusion, protein complex assembly, and cell motility. Membrane and cytoplasmic fractions were isolated from TM4 cell with or without testosterone administration. As shown in Figure 1(c), the expression of VAPA was unaltered in the input group after testosterone exposure. The binding of the protein to AR was decreased in the membrane fraction (*P* < 0.01) and increased in the cytoplasmic fraction under testosterone treatment (*P* < 0.01). These data indicated that VAPA may be involved in the AR membrane trafficking.

The article "Vesicle-Associated Membrane Protein-Associated Protein A Is Involved in Androgen Receptor Trafficking in Mouse Sertoli Cells" was retracted in 2019. Reasons: concerns about the data; concerns about the images; concerns about the results or conclusions.

### 3.2. VAPA Is Involved in AR Trafficking in Mouse Sertoli Cells

shRNA of VAPA was designed and synthesized to decrease the expression of VAPA in TM4 cell. Western blot and RT-PCR results in Figure 2(a) showed an effective knockdown of VAPA by the shRNA (*P* < 0.01). Cells transfected with negative control or VAPA shRNA were exposed to 10 nM testosterone for 30 min. Compared with the negative control, blots and data analysis showed a decrease in the membrane (1.00 ± 0.03 versus 0.55 ± 0.04, *P* < 0.05) and nuclear (1.00 ± 0.05 versus 0.69 ± 0.06, *P* < 0.05) localization at basal condition (Figures 2(b) and 2(c)). After exposure to testosterone, there were significant increases in membrane and nuclear proteins of both NC and shRNA group. However, AR trafficking to membrane in shRNA group (1.38 ± 0.08) was decreased, compared with the NC (0.67 ± 0.07, *P* < 0.01); and the nuclear trafficking was also inhibited (3.28 ± 0.34 versus 1.56 ± 0.18, *P* < 0.01).

### 3.3. VAPA-Mediated AR Trafficking via Vesicle Transport Protein OSBP

Experiments were conducted to study the molecular mechanism of AR trafficking mediated by VAPA. It was reported that VAPA interacts with OSBP (Oxysterol-binding protein) [8]. The expression of OSBP was unaltered in membrane and cytoplasmic fractions under testosterone treatment (Figures 3(a) and 3(c)). As shown in Figures 3(b) and 3(d), the binding of OSBP with AR was decreased in membrane fraction (1.00 ± 0.04 versus 0.42 ± 0.09, *P* < 0.01) but increased in the cytoplasmic fraction (1.00 ± 0.03 versus 2.21 ± 0.14, *P* < 0.01). The data analysis also showed that the association of VAPA and OSBP was increased in cytoplasmic fraction (1.00 ± 0.05 versus 1.35 ± 0.09, *P* < 0.05) but unchanged in membrane samples.

## 4. Discussion

Spermatogenesis is a complex and highly ordered process regulated by a series of gene products. Lots of clinical and experimental studies suggested that androgen and its receptor are critical for spermatogenesis and male fertility. Androgen controls spermatogenesis mainly by associating with the AR localized in Sertoli cells, and the role of androgen in Sertoli cells includes maintaining blood-testis barrier, meiosis, Sertoli-spermatid adhesion, and sperm release.

AR is capable of transmitting testosterone signals by at least 2 mechanisms, the classical and nonclassical pathways. In the classical signaling pathway, testosterone that diffuses through the cell membrane interacts with AR in the cytoplasm and then translocates to nucleus, binds AREs in gene regulatory regions, and recruits coactivator or corepressor proteins to regulate gene expression [9].

The article "Vesicle-Associated Membrane Protein-Associated Protein A Is Involved in Androgen Receptor Trafficking in Mouse Sertoli Cells" was retracted in 2019. Reasons: concerns about the data; concerns about the images; concerns about the results or conclusions.

In the nonclassical pathway, stimulation of Sertoli cells with levels of testosterone (10–250 nM) that are similar to or lower than that found in the testis causes a population of AR to localize near the plasma membrane. Studies using Western blot and immunofluorescence confirmed the localization of AR in membrane [10]. Binding of testosterone to AR allows the receptor to interact with and activate Src tyrosine kinase. Once activated, Src causes the phosphorylation of the epidermal growth factor receptor (EGFR) via an intracellular pathway, as well as kinase Ras. The stimulation of EGFR results in the activation of the MAP kinase cascade including the kinases RAF, MEK, and Erk [9]. In a previous study [6], we detected the membrane localization of AR, and testosterone induces AR translocation to membrane within 5 min (1.20 ± 0.02 fold change of basal value), the translocation was increased up to 60 minutes, and at 30-minute point, the fold change of AR translocation was 2.56 ± 0.02, then we choose 30 minutes treatment for further study.

In order to figure out the molecular mechanism of AR trafficking to membrane fraction, we identified the candidate proteins involved in this action using MS and bioinformatic analysis. 10 candidate proteins were identified; we conducted experiments to confirm the data and study the molecular mechanism mediating AR trafficking by these proteins.

VAPA is a vesicle membrane-associated protein, evolution conserved in species and participates the formation of lipid bilayer of the tight junction between endoplasmic reticulum and of other organelles. VAPA is a type IV membrane protein, localizes in the plasma membrane and intracellular vesicles [11]. It may also be associated with the cytoskeleton. This protein may function in vesicle trafficking, membrane fusion, protein complex assembly, and cell motility [12, 13]. It was reported that VAPA is involved in the regulation of several biological process by activation of the MAPK signaling pathway, including the activation of oncogenes, and the development of tumors [14]. VAPA may also facilitate the target protein to the plasma membrane [15]. Our data indicated that the association of AR to VAPA was decreased in membrane fraction and increased in cytoplasmic after exposure to testosterone. Knock down of VAPA decreases AR membrane and nuclear localization at basal condition prevented AR translocation to membrane or nucleus after testosterone treatment. These data indicated that VAPA is involved AR intracellular trafficking.

The article "Vesicle-Associated Membrane Protein-Associated Protein A Is Involved in Androgen Receptor Trafficking in Mouse Sertoli Cells" was retracted in 2019. Reasons: concerns about the data; concerns about the images; concerns about the results or conclusions.

VAPA has been shown to interact with the OSBP to modify export from the endoplasmic reticulum [8]. It is reported that this association is mediated by the FFAT motif in OSBP [16]. It is also reported that endosome endoplasmic reticulum contacts control actin nucleation and retromer function through VAPA-dependent regulation of phosphatidylinositol 4-phosphate (PI_4_P) [17]. The blots showed that the interaction of OSBP with AR or VAPA decreased in membrane fraction and increased in cytoplasmic after exposure to testosterone. This suggested that VAPA may mediate AR trafficking by interacting with OSBP.

## 5. Conclusions

In this study, we identified proteins involved in cytoplasmic AR translocation to plasma membrane under the treatment of testosterone at physiological concentration, and the data showed VAPA plays an important role in this process. Co-IP and Western blot results verified the MS analysis; further studies showed a decrease in AR membrane localization and trafficking in cells transfected with VAPA shRNA. AR trafficking in Sertoli cells might be mediated by VAPA via association with vesicle transport protein OSBP. This study is able to further enrich the molecular mechanism of the androgen actions in Sertoli cells and provide new insights into the nonclassical signaling pathway of testosterone, which mediate spermatogenesis.

## Figures and Tables

**Figure 1:** VAPA is identified as a candidate protein by MS. (a) Representative Western blots showed the cytoplasmic and membrane AR translocation in input samples and co-IP samples in TM4 cells. Data analysis from collected experiments (*n* = 5) showed a decrease of AR expression in cytoplasmic fraction and an increase in membrane. (b) Silver staining of the co-IP sample of the membrane proteins. The bands indicated by the dotted rectangle were subjected to mass spectrograph. (c) The film images showed the representative blots for AR and VAPA in membrane and cytoplasmic fractions, before (input) or after immunoprecipitation (co-IP) by the anti-AR antibody in TM4 cells treated with 10 nM testosterone for 30 min. For the input samples, data analysis from repeated experiment (*n* = 3) showed that VAPA expression was unchanged after exposure to testosterone. For the co-IP samples, the data indicated the association of VAPA and AR, which was showed as VAPA expression divided by AR expression. This experiment was repeated for three times. C: basal. T: 10 nM testosterone for 30 min. ^∗^*P* < 0.05; ^∗∗^*P* < 0.01.

**Figure 2:** VAPA is involved in AR trafficking. (a) Representative Western blot analysis and real-time PCR showed VAPA was knocked down by shRNA transfection. ^∗∗^*P* < 0.01, *n* = 3. (b) Representative Western blot analysis indicated that AR localization and trafficking in membrane and nuclear fractions were decreased in VAPA shRNA group. (c) Statistical analysis of collected data was from three repeated experiments. The left panel was for membrane fraction, and right for nucleus. The data was expressed as the fold change of AR expression level at basal condition in cells transfected with NC, and the data was showed as mean ± SEM. NC: cells transfected with the negative control vector. ^∗^*P* < 0.05; ^∗∗^*P* < 0.01.

The article "Vesicle-Associated Membrane Protein-Associated Protein A Is Involved in Androgen Receptor Trafficking in Mouse Sertoli Cells" was retracted in 2019. Reasons: concerns about the data; concerns about the images; concerns about the results or conclusions.

**Figure 3:** VAPA-mediated AR trafficking via vesicle transport protein OSBP. The film images showed the representative blots for AR, VAPA, and OSBP in membrane and cytoplasmic fractions, before (input, (a)) or after immunoprecipitation (co-IP, (b)) by the anti-AR antibody or anti-VAPA antibody in TM4 cells treated with 10 nM testosterone for 30 min. (c) The data analysis from three repeated experiments of panel (a). The data was expressed as the fold change of the OSBP expression in cytoplasmic fraction at basal condition, and the data was showed as mean ± SEM. (d) Collected data analysis showed the testosterone enhance AR and OSBP association, as well as the binding of VAPA and OSBP in cytoplasmic fraction, *n* = 4. The left panel was for the ratio of OSBP/AR (OSBP expression divided by AR expression) and the right for OSBP/VAPA (OSBP expression divided by VAPA expression). The data was expressed as the fold change of the values at basal condition, and the data was showed as mean ± SEM. ^∗^*P* < 0.05; ^∗∗^*P* < 0.01.

**Table 1:** Antibodies used in this study.

Antibody	Specie	Catalog	Dilution	Source
AR (N-20)	Rabbit	sc-816	1 : 1000	SCBT^∗^
Pan Cadherin	Mouse	ab22744	1 : 5000	Abcam
GAPDH	Goat	sc-23057	1 : 1000	SCBT^∗^
VAPA	Rabbit	ab96584	1 : 1000	Abcam
OSBP	Rabbit	GTX114602	1 : 1000	GeneTex

^∗^SCBT: Santa Cruz Biotechnology.
